The article "Regulation of somatostatin expression by vitamin D3 and valproic acid in human adipose-derived mesenchymal stem cells" was published in 2019. Journal: Stem Cell Res Ther.

# Regulation of somatostatin expression by vitamin D3 and valproic acid in human adipose-derived mesenchymal stem cells

**DOI:** 10.1186/s13287-019-1330-x

**Published:** 2019-08-06

**Authors:** Luise Doering, Rahul Khatri, Sebastian Friedrich Petry, Heinrich Sauer, Hans-Peter Howaldt, Thomas Linn

**Affiliations:** 1 Clinical Research Unit, Centre of Internal Medicine, Justus Liebig University, Friedrichstrasse. 20/ Aulweg 123, 35392 Giessen, Germany; 2 Institute of Physiology, Justus Liebig University, Giessen, Germany; 3 Department of Oral and Maxillofacial Surgery, University Hospital of Giessen and Marburg, Klinikstrasse. 33, 35392 Giessen, Germany

**Keywords:** Human adipose-derived mesenchymal stem cells, Somatostatin expression

## Abstract

**Background:**

Adipose-derived mesenchymal stem cells (ADMSC) are non-haematopoietic, fibroblast-like multipotent progenitor cells. They have the potential for trilineage (adipocyte, chondrocyte and osteocyte) differentiation as well as differentiation into endocrine pancreatic progenitors. In diabetic or cancer therapy, somatostatin (SST) expression plays a vital role. Small molecules such as valproic acid (VPA) and micronutrients like vitamin D3 have differentiation potential in ADMSC. Therefore, the aim of this study was to investigate the role of vitamin D3 machinery and its metabolic enzymes in ADMSC. Furthermore, the reprogramming effect of vitamin D3 and VPA was evaluated on somatostatin expression in pancreatic lineage differentiation.

**Methods:**

ADMSC were characterised based on their cell surface marker profile using flow cytometry. Specific adipogenic and osteogenic differentiation protocols were used in this study. Gene expression of several pluripotent, endodermal, pancreatic progenitor and pancreatic endocrine lineage markers were investigated in native ADMSC and after stimulation with different concentration of vitamin D3 for five consecutive days (0, 50, 100, 150 nM) and VPA (0.5, 1, 1.5, 2 mM) by real-time PCR. Furthermore, somatostatin expression was confirmed with ELISA and immunocytochemistry.

**Results:**

In ADMSC, the expression of somatostatin mRNA, the vitamin D receptor (VDR) and its metabolising enzymes 1 α-Hydroxylase, 24-Hydroxylase and 25-Hydroxylase were detected. Upon stimulation with vitamin D3, nuclear translocation of vitamin D receptor (VDR) was observed. Interestingly, the presence of vitamin D3 reduced the transcription of the somatostatin gene. By contrast, VPA treatment of cultivated ADMSC showed enhancing effect on somatostatin gene expression. No other pluripotent, endodermal, pancreatic progenitor or pancreatic endocrine lineage mRNA expression was modulated under the influence of vitamin D3 and VPA.

**Conclusion:**

Human ADMSC carry the VDR. The vitamin D metabolising enzyme 25-Hydroxylase responded to the addition of vitamin D3. Moreover, our results demonstrate that somatostatin expression in ADMSC is constitutive, partially secreted and regulated by vitamin D3 and VPA.

## Background

The endocrine pancreas harbours hormones from the pancreatic islets of Langerhans, comprised of several cell types: β-cells secrete insulin, α-cells secrete glucagon, δ-cells secrete somatostatin, PP cells secrete pancreatic polypeptide and ε-cells secrete ghrelin [1, 2]. A disturbance in the insulin metabolism leads to diabetes mellitus. Type 1 diabetes mellitus is characterised by an autoimmune destruction of β-cells and results in absolute insulin deficiency. Type 2 diabetes mellitus starts off with a reduced action of insulin, which subsequently leads to a deficient insulin secretion and reduction of β-cell mass as well [3–5]. Strategies have been developed to restore β-cell function, such as pancreatic islet transplantation, but inadequate donor and immunosuppression restrict its application [6]. Pluripotent stem cells are considered as a novel source for insulin-producing β-like cells or pancreatic progenitors cells to correct hyperglycaemia [7]. However, ethical and safety issues hamper the application of pluripotent stem cells [8, 9]. In this regard, mesenchymal stem cells (MSC) are non-haematopoietic, fibroblast-like multipotent stromal cells having potential to differentiate into trilineage, Schwann cells and endocrine lineage in vitro [10–14]. However, more effective and reproducible protocols involving media fortified with specific small molecules and micronutrients are required to overcome issues regarding differentiation. The impact of small molecules, such as valproic acid (VPA) and micronutrients like vitamin D3 on osteogenic differentiation of human MSC was studied, revealing a pro-differentiation potential [15, 16].

The prohormone vitamin D3 (cholecalciferol) with its active forms calcifediol (1α, 25(OH)_2_D_3_) and calcitriol (1α, 25-dihydroxyvitamin D_3_) regulates intestinal and renal absorption of calcium and phosphate [17]. It triggers both osteoclasts and osteoblasts, thus promoting bone regeneration and formation. Vitamin D3 deficiency leads to rickets in childhood [18] and is also associated with prostate, colon and breast cancer; inflammation; and diabetes mellitus [19–22]. Vitamin D supply is covered either by food consumption or conversion of 7-dehydrocholesterol by ultraviolet light in the skin which finally binds to vitamin D binding protein. In the liver, 25-Hydroxylase converts cholecalciferol into 25(OH)D_3_, which is turned into 25(OH)_2_D_3_ in the kidney by 1α-Hydroxylase (CYP27B1). Excessive calcitriol is converted into an inactive form via 24-Hydroxylase (CYP24A1) and removed in the form of calcitroic acid from the body [23]. The interaction of vitamin D3 and its receptor VDR has been studied in cardiomyocytes, vascular smooth muscle and endothelial cells [24–26], but the interaction in human MSC has not yet been elucidated.

Valproic acid (VPA) is a short-chain fatty acid with inhibiting effects on histone deacetylases in cell culture [27]. Moreover, it is a licenced drug in neurological conditions, such as epilepsy and migraine prophylaxis [28–32]. In addition, VPA was recently reported to modulate neurogenic, hepatogenic and osteogenic differentiation of MSC [16, 33, 34]. However, the mechanism of VPA in MSC differentiation towards pancreatic lineage was not examined so far.

Somatostatin (SST) is a peptide hormone expressed in the highest quantity in the gastrointestinal tract including the pancreas, but also the central nervous system. One of its known functions is in the interplay of endocrine pancreatic hormones, as it inhibits both insulin and glucagon secretion [35]. Moreover, it reduces the activity of other secretory types of cells, such as the parietal cells of the stomach and gastrin-producing cells, thereby slowing down the motility of the small bowel.

SST has two active forms produced by alternative cleavage of a single preproprotein: one of 14 amino acids and the other of 28 amino acids. Human SST gene is one out of six known in vertebrates. In conjunction with the five somatostatin receptors, SST possesses a large range of functions.

In this study, we first characterised primary adipose tissue-derived mesenchymal stem cells (ADMSC) to test the capacity of osteogenic and adipogenic differentiation as well as constitutive expression of selected genes of the endocrine pancreas. Second, vitamin D machinery, VDR and its metabolising enzymes were confirmed. Third, we exposed ADMSC to vitamin D3 and VPA with the idea that the expression of one or more pancreatic genes was changed in a significant way. Interestingly, we found that somatostatin was the single endocrine marker highly expressed in ADMSC and was significantly regulated on both mRNA and protein level by vitamin D3 and VPA.

## Material and methods

### Human adipose-derived stem/stromal cells (ADMSC) isolation and cell culture

Cells were isolated from subcutaneous fat as described [36, 37]. Briefly, adipose tissue was separately dissected into small pieces, transferred into a sterile blood bag and treated with washing steps for 2 h using phosphate-buffered saline and adding 0.075% Liberase™ (Roche, Mannheim, Germany) for enzymatic digestion. After centrifugation, the harvested cells were seeded into 75-cm^2^ tissue culture flasks containing Ham’s F-10 medium supplemented with 10% foetal calf serum (FCS; Sigma, Deisenhofen, Germany), 2 mM glutamine, 0.1 mM β-mercaptoethanol, 2 mM minimal essential medium, 100 IU/ml penicillin and 100 μg/ml streptomycin (Invitrogen, Karlsruhe, Germany) and placed in an incubator (5% CO_2_, humidified air at 37 °C). Within 10 days of culture, cells attained confluency and a fibroblast-like appearance. For further cultivation, an expansion medium, containing DMEM (4500 mg Glc/l) medium supplemented with 19.95% heat-inactivated FCS (Sigma, Deisenhofen, Germany), 1% glutamine, 1% non-essential-amino acids and 0.39% penicillin/streptomycin (Invitrogen, Karlsruhe, Germany), was used. In all experiments, ADMSC were cultivated up to passage eight.

### MSC marker profiling and differentiation

ADMSC were cultivated and harvested with trypsin-EDTA (Life Technologies, Germany). Enzymatic reaction of trypsin-EDTA was stopped with DMEM containing 20% FCS. Cells were washed twice, stained for MSC markers CD90^+^, CD44^+^, CD105^+^ and CD44^+^ (BD Stemflow™; Germany) and were analysed by flow cytometry (FACS Canto, BD). To demonstrate the differential pattern of the ADMSC towards adipogenic and osteogenic lineage, the StemPro® Adipogenesis and the Osteogenesis Kit (Life Technologies, Germany) were utilised.

### Vitamin D3 and valproic acid (VPA) treatment of ADMSC

1 × 10^6^ cells were cultured according to the above-mentioned conditions in the absence and presence of increasing concentrations (0 nM, 50 nM, 100 nM, 150 nM) of vitamin D3 for five consecutive days. Similarly, 1 × 10^6^ cells were treated with VPA (0.5 mM, 1 mM, 1.5 mM, 2 mM) for five consecutive days. Afterwards, cells were harvested and analysed with a Western blot and real-time polymerase chain reaction (PCR) (Thermo Fisher Scientific, Germany).

### Western blot

ADMSC cell lysates were prepared using buffer customised for immunoprecipitation containing protease inhibitors (RIPA, Cell Signaling Technology, Germany). Cytoplasmic and nuclear fractions were prepared with NE-PER nuclear and cytoplasmic extraction reagent (Thermo Scientific, Cat-No-78833) in accordance with the manufacturer’s protocol. Protein concentration was measured with Bradford assay (Bio-Rad, Germany). Samples were mixed with Laemmli buffer (Carl Roth, Germany) and 20% β-mercaptoethanol (Life Technologies, Germany) and denatured for 5 min at 95 °C. Proteins were separated with sodium dodecyl sulphate polyacrylamide gel electrophoresis followed by transfer to activated polyvinylidene difluoride membrane. Membranes were washed with Tris buffered containing Tween 20 for 5 min and blocked with 5% skimmed milk solution for 1 h to block non-specific protein binding. The membrane was incubated overnight at 4 °C on rocker with monoclonal VDR rabbit anti-human antibody from Epitomics (Cat-No 3277-1) diluted 1:1000, β-tubulin (Abcam; 1:10,000 Cat-No, ab52623) and Lamin A/C (Gentex; 1:2000, Cat-No GTX111677). The membrane was washed again three times. Secondary antibody goat anti-rabbit Ig-HRP from Dako (Cat-No.-P0448) in 1:3000 dilution was added for 1 h at room temperature. After three washes, membranes were incubated with enhanced chemiluminescence solution for 1 min and film was developed with Odyssey® imaging system (LICOR®, Germany).

### Quantitative real-time polymerase chain reaction (qRT-PCR)

RNA was isolated with Qiagen RNA isolation kit (Qiagen, Germany). RNA quantification was performed using a NanoDrop spectrophotometer (NanoDrop, USA). One thousand nanograms of RNA was reverse transcribed to synthesised cDNA with SuperScript III (Invitrogen, USA). Real-time PCR was accomplished with 20 μl reaction aliquots containing SYBR Green (Bio-Rad Laboratories, Germany), specific primers, cDNA template and water. PCR comprised of the following conditions: denaturation (95 °C, 10 min) followed by 40 cycles at 95 °C for 10 s, 60 °C for 20 s and 72 °C for 10 s. Target gene expression was normalised with the housekeeping gene or HPRT gene and calculated with the 2^ΔΔCt^ method. All primers (Table 1) were designed and tested for their specific sequence by primer blast.

**Table 1:** Primers

1 HPRT	Forward	TCAGGCAGTATAATCCAAAGATGGT
	Reverse	AGTCTGGCTTATATCCAACACTTCG
2 c-kit	Forward	GGCATCACGGTGACTTCAAT
	Reverse	GGTTTGGGGAATGCTTCATA
3 Thy1	Forward	ATGAAGGTCCTCTACTTATCCGC
	Reverse	GCACTGTGACGTTCTGGGA
4 SCF	Forward	GGTGGCAAATCTTCCAAAA
	Reverse	TCTTTCACGCACTCCACAAG
5 SST	Forward	GATGCCCTGGAACCTGAAGA
	Reverse	CCGGGTTTGAGTTAGCAGATCT
6 VDR	Forward	CCAGTTCGTGTGAATGATGG
	Reverse	GTCGTCCATGGTGAAGGA
7 1 α-Hydroxylase	Forward	TGTTTGCATTTGCTCAGA
	Reverse	CCGGGAGAGCTCATACAG
8 24-Hydroxylase	Forward	GCAGCCTAGTGCAGATTT
	Reverse	ATTCACCCAGAACTGTTG
9 25-Hydroxylase	Forward	GGCAAGTACCCAGTACGG
	Reverse	AGCAAATAGCTTCCAAGG
11 Insulin	Forward	GCAGCCTTTGTGAACCAACA
	Reverse	TTCCCCGCACACTAGGTAGAGA
12 PDX-1	Forward	TGATACTGGATTGGCGTTGTTT
	Reverse	TCCCAAGGTGGAGTGCTGTAG
13 Glucagon	Forward	CCCAAGATTTTGTGCAGTGGTT
	Reverse	CAGCATGTCTCTCAAATTCATCGT
14 NeuroG3	Forward	CTATTCTTTTGCGCCGGTAGA
	Reverse	CTCACGGGTCACTTGGACAGT
15 Nestin	Forward	CGTTGGAACAGAGGTTGGAG
	Reverse	TAAGAAAGGCTGGCACAGGT

### Immunocytochemistry

To examine the protein distribution within the cells, immunocytochemistry was performed. Cells were cultured on glass slides (Superfrost Ultraplus, Langenbrinck, Germany). After treatment with vitamin D3 (5 min, 10 min, 30 min) and VPA (1 mM for five consecutive days), ADMSC were fixed with 4% paraformaldehyde. Cells were permeabilised for 10 min with 0.1% PBS-T followed by blocking (PBS; 1% donkey serum and Triton X-100 (0.2%)) for 20 min at room temperature. Primary antibodies, i.e. rabbit anti-VRD (1:200) and rabbit anti-somatostatin (1:100), were incubated overnight at 4 °C. Next day, slides were washed with PBS and stained for secondary antibodies: fluorescein FITC donkey-anti-Rabbit (1:400), donkey-anti-rabbit rhodamine red (1:400) in PBS containing 0.01% PBS-T and 5% human-serum. Slides were washed twice, and nuclear staining was performed with Hoechst (Calbiochem, Germany). Slides were washed once and fixed with Prolong Gold (Invitrogen, Germany). Pictures were captured with DM6000B florescent microscope (Leica, Germany).

To investigate the differentiation of ADMSC into adipocyte-like and osteocyte-like cells, slides were fixed with formalin (Fischer, Germany) for 30 min. ADMSC cultivated on glass slides were washed with ethanol (50%) and stained with Sudan III (Sigma, Germany) at room temperature for 35 min to find lipid droplets. Counterstain was performed with hemalum (Merck, Germany). Osteocyte-like cells were identified by incubating with alizarin red for 4 min, washed with water and counterstained with trypan blue (Sigma, Germany).

The translocation of the VDR into the nucleus was quantified by analysing respective images from immunocytological staining with ImageJ (Wayne Rasband, National Institutes of Health, USA). Briefly, ImageJ was calibrated to match the scale of the respective image. For each cell, the freehand tool was then used to roughly select an ROI containing the nucleus on the channel filtered for nuclei (DAPI/blue). A threshold value was then employed to precisely select the nucleus and measure its area. The nucleic outline was saved as a new ROI and transferred to the channel filtered for VDR staining (FITC/green). The VDR staining inside the nucleic ROI was consecutively selected using a threshold value to avoid inclusion of unspecific background staining. The nucleic VDR staining area was then measured and divided by the respective nucleic area for normalisation.

### Enzyme-linked immunosorbent assay (ELISA)

#### Cultivation protocol

To investigate the regulation of synthesis and secretion in ADMSC, an enzyme-linked immunosorbent assay of human somatostatin was applied. For this purpose, ADMSC were cultured in 5-ml media per well. Samples from supernatant and cells were collected at 0, 24, 48, 72 and 120 h of cultivation 1 h after medium change. In separate experiments with the histone deacetylase inhibitor VPA, cells were grown in 24-well plates (Cellstar, Greiner Bio-One GmbH, Frickenhausen, Germany) and cultured in the absence or presence of increasing concentrations of VPA (0.25, 0.5, 1, 1.5 and 2.0 mM).

#### Analysis of somatostatin (SST)

Protein concentrations were determined by Bradford assay. A biotinylated rabbit anti-human antibody captured the N-terminus of pro-SST (25–116) (EIAab, antikörper-online GmbH, Aachen, Germany). Briefly, 100 μl avidin-conjugated horseradish peroxidase was added to 100 μl sample using microplate and incubated for 45 min at 37 °C. Subsequently, 90 μl tetramethylbenzidine was added, and while protected from light, the plate was incubated for 20 min at 37 °C. The reaction was finalised with 50 μl stopping solution with sulphuric acid, and readings were performed at 450 nm using a multimode reader (Mithras, Berthold, Germany).

#### Calculations

The secretion rate per hour was calculated from SST levels measured in samples of culture medium. SST is initially secreted as a 116-amino acid precursor, which undergoes endoproteolytic cleavage of the signal peptide resulting in pro-SST (25–116) with a molecular weight of 10.3 kDa. Pro-SST (25–116) may be processed into two active forms, SST-14 (103–116) and SST-28 (89–116). The minimal detectable concentration of SST (25–116) was 9.7 pmol/l. The standard curve was constructed from six levels of solutions between 0 and 2.4 pmol/l. Coefficients for intra- and inter-assay variations were less than 10%. Results were normalised to protein concentrations resulting in pmol SST per mg protein.

### Statistical analysis

Graph Pad Prism 6 (GraphPad Software, San Diego, CA, USA) was utilised for statistical analysis. Skewed data sets were log-transformed to ensure normal distribution. One-way ANOVA and Student’s *t* test were performed for most of the statistics unless otherwise stated. Data are represented as mean values ± SEM with *n* reflecting the number of experiments. *p* < 0.05 was considered significant (*p < 0.05, **p < 0.01, ***p < 0.001).

## Results

### Characterisation of ADMSC

#### Cell surface marker profile

ADMSC were characterised based on their cell surface marker profile by flow cytometry. In Fig. 1a, the upper panel depicts the control for the respective population. As presented in the lower panel, sample cells were double positive for CD90^+^ and CD44^+^ (98.9%), CD105^+^ and CD44^+^ (98.7%) and CD73^+^ and CD44^+^ population (97.8%).

**Fig. 1:** Characterisation and differentiation of ADMSC. **a** Flow cytometry analysis of ADMSC surface marker profiling. Cells were stained and characterised based on CD90^+^, CD44^+^, CD105^+^ and CD73^+^ markers using flow cytometry, and plots were analysed with FACSDiva software. **b** ADMSC were cultivated on glass slides for 5 days using adipogenic culture medium. Slides were washed with 50% ethanol, and intracellular fat vacuoles were stained red with Sudan III (arrow) following treatment with adipogenic (**b** (1)) or regular (**b** (2)) medium. Magnification × 200. **c** The conversion of ADMSC into osteoblast-like cells was demonstrated cultivating them with osteogenic medium. **c** (1) shows ADMSC cultivated with regular medium, **c** (2) and **c** (3) cultivated with osteogenic medium for 5 days. Osteoblast-like cells were identified using alizarin red, and images were captured with a light microscopy Leica microsystem ICC50 HD. For **c** (1) and **c** (3), × 200 magnification and, for **c**2, × 50 magnification were considered

#### Adipogenic differentiation

After 1 week of culture in adipogenic medium, ADMSC enlarged and started differentiating into adipogenic lineage. Two weeks onward, the first fat vacuoles were observed. After 17 days, more than 50% of the cells were positive for Sudan III as shown in Fig. 1b. When ADMSC were cultivated in normal expanding culture medium, fat vacuoles remained absent throughout.

#### Osteogenic differentiation

One week of osteogenic medium resulted in ADMSC becoming rounder and smaller. Subsequently, ADMSC differentiation into osteocyte-like cells was confirmed with alizarin red and methylene blue staining as shown in Fig. 1c. The control was subjected to expanding medium. Only ADMSC maintained in osteogenic medium, but not those cultivated in regular medium clearly showed intra- and extracellular calcium deposits.

### mRNA expression of native ADMSC

Expression of gene transcripts associated with pluripotency (c-kit, Thy1, Nanog, Sox2, Oct4, SCF), endoderm (CXCR4, FoxA2, Nestin, Sox17), pancreatic duct (Pdx1, NeuroG3, Nestin), pancreatic endocrine cells (insulin, glucagon and somatostatin (SST)), transcripts of vitamin D3 receptor and its metabolising enzyme genes were investigated. HPRT was selected as an unregulated housekeeping gene. With normal cell culture medium, RNA products of Thy1, c-kit, SCF, SST, VDR, 1 α-Hydroxylase, 24-Hydroxylase and 25-Hydroxylase were detected by qRT-PCR (Fig. 2a) and on agarose gel as well (data not shown). No transcripts were observed for all of the other genes from the list. Next, we examined whether VDR protein was constitutively synthesised at the basal level. Western blot showed a clear band at 54 kDa, confirming VDR expression (Fig. 2b).

**Fig. 2:** **a** Significant constitutive transcription of HPRT, Thy1, SCF, c-kit, somatostatin (SST), VDR and vitamin D machinery enzymes (1α-Hydroxylase, 24-Hydroxylase and 25-Hydroxylase) out of a total panel of 15 genes were detected at normal culture conditions of ADMSC. **b** Western blot gel was loaded with 40 μg (lane 1) and 20 μg (lane 2) of ADMC lysate. The 54 kDa vitamin D receptor (VDR) protein was probed with a monoclonal rabbit anti-human antibody followed by goat anti-rabbit Ig-HRP secondary antibody. The membrane was incubated with enhanced chemiluminescence solution for 1 min and developed with Odyssey® imaging system (LICOR®, Germany). For PCR analysis, HPRT was considered as a housekeeping gene and fold change was achieved with 2^−∆∆Ct^ method. To compare the groups, one-way ANOVA with Turkey’s post hoc test was utilised

### Effect of vitamin D3 on gene expression of ADMSC

ADMSC differentiation potential towards endocrine lineage was assessed with increasing concentrations of vitamin D3 (50, 100, 150 nM). However, no significant difference was observed in the pluripotent (c-kit, Thy1, Nanog, Sox2, Oct4, SCF), endoderm (CXCR4, FoxA2, Nestin, Sox17), pancreatic duct (Pdx1, NeuroG3, Nestin) and pancreatic endocrine (insulin, glucagon) markers at the transcript level (data not shown) except for somatostatin (SST). Furthermore, vitamin D3-related hydroxylases were analysed. Significant increment of 24-Hydroxylase at the transcript level was observed upon vitamin D3 stimulation compared to the absence of vitamin D3 (Fig. 3d). No change was observed in the mRNA expression of VDR, 1α-Hydroxylase and 25-Hydroxylase (Fig. 3a–c). Interestingly, a significant downregulation of SST transcription was observed. At 50 nM vitamin D3, the relative expression of somatostatin decreased to 69.5 ± 5.9% (*p* < 0.01) and declined further at 100 nM to 34.5 ± 10.6% (*p* < 0.001). Upon exposure to 150 nM vitamin D3, relative mRNA expression marginally increased again as demonstrated in Fig. 3e.

**Fig. 3:** Influence of increasing concentrations (50, 100, 150 nM) of vitamin D3 to 120 h culture of ADMSC on the expression of selected gene transcripts. **a–d** The influence of vitamin D3 on the gene expression levels of metabolising enzymes 1α-Hydroxylase, 24-Hydroxylase, 25-Hydroxylase and the VDR. The expression of 24-Hydroxylase was regulated by vitamin D3 compared to control without vitamin D3 (*p* < 0.001) while other target gene transcripts remained stable without changes. **e** Relative expression of somatostatin gene was modulated in decreasing fashion in the presence of vitamin D3 (*p* < 0.001). Data represent the mean ± SEM (*n* = 4 runs). To compare the different concentration, one-way ANOVA with Turkey’s post hoc test was utilised. Values considered significant *p < 0.05, **p < 0.01 and ***p < 0.001, compared with the absence of vitamin D3 as a control condition

### Stimulation of VDR receptor by vitamin D3

When ADMSC were stimulated with vitamin D3, nuclear translocation of the VDR could be detected in and out of the nucleus. In the absence of vitamin D3, the VDR was observed in the cytoplasm as shown in Fig. 4a at 0 min. After the addition of vitamin D3, within 5 min of VDR stimulation, granules were formed around the nucleus. Ten minutes later, nuclear accumulation of the VDR was observed. Nuclear accumulation of the VDR was enhanced with time (30 min) as shown in Fig. 4a. Quantification of the nuclear VDR content confirmed the optical impression. In comparison with untreated control cells, the amount of the VDR in the nucleus area was significantly increased after 10 min (*p* < 0.05) and 30 min (*p* < 0.005, Fig. 4b). Further, Western blot was performed with different fraction of the ADMSC after stimulating with vitamin D3 at different time points. At 0 min, VDR bands at 54 kDa were observed in the cytoplasmic (1) and nuclear fraction (2) as shown in Fig. 4c. After 5 min, VDR started accumulating in the nucleus from the cytoplasm. VDR shift to the nuclear fraction was observed after 10 min and 30 min as shown in Fig. 4c. β-tubulin (52 kDa) and lamin A/C (74 kDa) were considered as a positive control for cytoplasmic and nuclear fraction.

**Fig. 4:** Representative images of VDR translocation from cytoplasm to nucleus observed in the presence of 100 nM vitamin D3 and the respective quantification. **a** The time-dependent movement of VDR, without vitamin D3 at 0 min, 5 min, 10 min and 30 min of vitamin D3 addition, translocation from cytoplasm to nucleus was observed. Arrows point to VDR-positive cell structures either in the cytoplasm (broad) or nucleus (narrow arrow). **b** Quantification of the VDR translocation. Nucleic VDR staining area was normalised by division with the respective nucleus’s area. Comparison of the VDR/nucleic area ratio between vitamin D3-treated cells and untreated controls by ANOVA confirmed the optical impression of the significant shift of the VDR into the nucleus. **c** The Western blot of VDR time-dependent translocation from the cytoplasm (1) to nucleus (2) post addition of vitamin D3 at 0 min, 5 min, 10 min and 30 min. β-Tubulin (52 kDa) and lamin A/C (74 kDa) were considered as a positive control for cytoplasmic and nuclear fraction. Data represent mean ± SEM (*n* = 19–47 cells per time point); 1, cytoplasmic fraction; 2, nuclear fraction, **p < 0.005, *p < 0.05

### Effect of histone deacetylase inhibitor valproic acid (VPA) on ADMSC

When ADMSC were treated with VPA, no upregulation of the endocrine markers (pluripotent, endoderm, pancreatic duct and pancreatic endocrine) were detected (data not shown) except for somatostatin. SST gene transcription was significantly increased (3.6 ± 0.3, fold, *p* < 0.001) in the presence of 1 mM VPA as compared with the untreated control (Fig. 5a). Pro-SST (25–116) was expressed in cultivated ADMSC. Interestingly, pro-SST was also released to the culture medium. Our experimental design allowed to calculate the quantities of secreted pro-SST ranging from 0.26 ± 0.03 to 0.44 ± 0.06 pmol/mg/h (Fig. 5b (1)). The variability of extracellular transport during culture time up to 120 h was not significant (*p* = 0.116). Mean pro-SST secretion rate at all time points was 0.33 ± 0.10 pmol/mg/h. Cells accumulated 25.3 ± 3.4 pmol SST (25–116) per mg protein within 120 h of culture, and they excreted 52% (13.1 ± 1.7 pmol/mg) of the total amount.

**Fig. 5:** Effect of valproic acid (VPA) on somatostatin (SST) production and secretion of ADMSC. **a** SST mRNA expression was increased 3.6 ± 0.3 fold by 1 mM VPA after 5 days of culture compared to the absence of VPA (*n* = 5, *p* < 0.001). **b** (1) Pro-SST protein was released to the culture medium. An aliquot of the supernatant was sampled 24 h after medium change for each time point. SST 25–116 peptide concentrations were measured by Elisa as described in the ‘Materials and methods’ section normalised to the protein content (mg) of the supernatant. Secretion was calculated from three independent experiments at five time points (0, 24, 48, 72 and 120 h) of ADMSC cultivation. Cells were cultured in 5-ml media per well, and secretion rates were given in pmol SST 25–116 per mg protein an hour. **b** (2) Cellular SST 25–116 production was upregulated by VPA added at 0, 0.25, 0.5, 1, 1.5 and 2.0 mM final concentrations. Analysis of variance resulted in significant difference (*p* = 0.008). **b** (3) SST 25–116 production in response to VPA concentration was plotted. Data were fit to a non-linear function with the assumption that intracellular SST 25–116 was increased by the presence of VPA in the medium of cultivated ADSC. Half-maximal effective concentration of VPA to stimulate SST synthesis was 0.4 mM (*R*^2^ = 0.79). **c** Staining of ADMSC with rabbit anti-somatostatin antibody. **c** (1) ADMSC cultivated in normal medium showed aggregates of SST within the cytoplasm. **c** (2) Cultivation in the presence of 1 mM VPA for 120 h resulted in higher density of aggregates adjacent to cell membrane. For PCR analysis, HPRT was considered as a housekeeping gene and fold change was achieved with 2^−∆∆Ct^ method. To compare the groups, one-way ANOVA with Turkey’s post hoc test was utilised. Data represent the mean ± SEM. *p < 0.05, **p < 0.01, ***p < 0.001 versus control condition without VPA

When VPA was added to ADMSC in culture, there was a 65% increase of cellular SST (25–116) production compared to control (0 VPA, 44.7 ± 3.4) at 1 and 1.5 mM VPA (73.3 ± 3.8 and 73.6 ± 3.6 pmol/mg, *p* < 0.01), respectively (Fig. 5b (2)). The secreted total fraction was constant within a range of 40–49% as secretion rates increased accordingly to cellular production from 0.86 ± 0.13 pmol/mg/h (0 VPA, control) to 1.25 ± 0.03 pmol/mg/h (1 mM VPA). Data were fitted using semi-logarithmic plot of cellular SST (25–116) content in response to VPA concentrations which resulted in half-maximal effect of SST release at 0.4 mM VPA (Fig. 5b (3)).

### Modification of cellular SST under the influence of VPA

Adherent ADMSC were examined with an immunofluorescent microscope using rabbit anti-SST antibody and rhodamine red secondary antibody. Cytoplasmic compactions of SST staining were observed (Fig. 5c (1)). In the presence of 1 mM VPA, they were increased in number and gathered at the cell membrane (Fig. 5c (2)).

## Discussion

In this study, the oligopotent character of ADMSC was demonstrated by differentiation into the osteogenic and adipogenic cell lineage. Cells were confirmed for their plastic adherence and fibroblast-like appearance. They expressed distinguished MSC markers CD90^+^, CD44^+^, CD105^+^ and CD73^+^ and were negative for haematopoietic lineage, thereby fulfilling the criteria of International Society Cell and Gene Therapy. Transcripts indicating endodermal or pancreatic differentiation were not expressed in cultivated ADMSC.

The pluripotential capacity of the ADMSC was confirmed by the expression of SCF, c-kit and Thy1. Since higher passages were reported to wield reduced Thy1 expression, only passages two to eight were employed in the current study. As expected, Thy1 expression proved to be constant during these successive passages.

Vitamin D was reported to upregulate VDR and 24-Hydroxylase and downregulate 1 α-Hydroxylase in porcine ADMSC [23]. Moreover, human MSC were investigated in the context of bone reconstitution under the influence of vitamin D3 [38]. Our study confirmed that human ADMSC possess both receptor and enzymes required for full vitamin D synthesis. After the addition of vitamin D3 to MSC culture, a nuclear shift of the VDR along with higher 24-Hydroxylase expression was observed. Previously, human genetic studies linking vitamin D and VDR to diabetes mellitus suggested a potential role in pancreatic β-cell cycle and survival [39]. VDR was reported to be expressed in human foetal pancreatic progenitor cell, and proliferation of these cells was modulated by vitamin D [40]. Recently, a VDR-dependent transcriptional programme was reported in induced pluripotent stem cell lines harbouring inducible small hairpin RNA knockdowns of VDR. They differentiated into β-cells like cells via a complex of VDR and bromodomain proteins BRD 7 and 9 [41]. In addition, vitamin D and its analogs suppressed Wnt signalling which was identified as an essential pathway in the differentiation of β- and δ-cells alike by repressing beta-catenin/TCF-4 transcriptional activity [6, 42, 43].

Somatostatin acts via a G-protein-coupled specific receptor on cells to regulate synthesis and release of proteins, such as growth hormone, glucagon and insulin. Human adipocytes were reported to release several peptides, including somatostatin, with a major impact on the immune response and glucose metabolism [44–46]. Somatostatin expression and its receptor are present in inflamed adipose tissue of septic disease patients [47].

Our data from primary ADMSC confirmed constitutive somatostatin expression, which was downregulated in the presence of vitamin D3 in cell culture. Biosynthesis and release of somatostatin and other neuropeptides are known to be regulated by the second messenger cyclic adenosine monophosphate. The activator forskolin induced somatostatin gene transcription eight- to tenfold and required the 30-nucleotide response element of cyclic adenosine monophosphate [48]. Conversely, the addition of 1,25-vitamin D reduced second messenger-regulated transcription of somatostatin [49, 50].

Apart from the regulation by vitamin D3, the VPA’s effect on SST synthesis was published in regard to neurogenic and osteogenic differentiation of MSC [51, 52]. Furthermore, VPA treatment supported β-cell viability and proliferation, thereby ameliorating hyperglycaemia in diabetic rats [43, 44]. VPA was further reported to inhibit histone deacetylase (HDAC) class I and II activity and to induce specific degradation of histone deacetylases in the proteasome [53, 54]. Histone deacetylase inhibitors were demonstrated to modify timing and determination of pancreatic cell fate [55]. Analyses of the pancreas of class IIa HDAC mutant mice revealed an increased pool of somatostatin-producing δ-cells. Treatment of pancreatic explants with class IIa HDAC inhibitor enhanced expression of Pax4, a key factor required for both proper β- and δ-cell differentiation [56]. Therefore, we investigated VPA’s potential as a modulating drug of the somatostatin machinery. VPA presence in the medium increased pro-SST on the secreted and intracellular level of cultured ADMSC. Interestingly, the formation of somatostatin aggregates was noticed in the cytoplasm by immunofluorescent staining of adherent ADMSC in culture. However, no other differentiation potential towards endodermal or pancreatic progenitor markers were detected.

## Conclusions

Taken together, our study demonstrates that primary human ADMSC were capable of regulating the production and release of SST. Downregulation was achieved with vitamin D3 and upregulation with VPA. Switching on or off the SST machinery in ADMSC should be further investigated in vivo in preclinical models of diabetes mellitus.

## Data Availability

All relevant data and material to reproduce the findings are available in the manuscript.

## Abbreviations

ADMSC: Adipose-derived mesenchymal stem cells
ANOVA: Analysis of variance
cDNA: Complementary deoxyribonucleic acid
c-kit: Proto-oncogene receptor tyrosine kinase
Ct: Threshold cycle
CXCR4: C-X-C chemokine receptor type 4, synonym CD184
DM: Diabetes mellitus
DMEM: Dulbecco’s modified Eagle’s medium
Elisa: Enzyme-linked immunosorbent assay
FCS: Foetal calf serum
FITC: Fluorescein isothiocyanate
FoxA2: Forkhead box protein A2
mRNA: Messenger ribonucleic acid
MSC: Mesenchymal stem cells
Nanog: Tir na nOg (Irish, ‘Land of the Young’), homeobox protein transcription factor
Nestin: Neuroectodermal stem cell marker
Oct4: Octamer binding transcription factor
PBS: Phosphate-buffered saline
qRT-PCR: Quantitative real-time polymerase chain reaction
SCF: Stem cell factor
SEM: Standard error of the mean
Sox17: SOX (SRY-related HMG-box) family of transcription factors
Sox2: Sex-determining region Y (SRY)—box 2
SST: Somatostatin
synonyms CD 117: Stem cell factor receptor
Thy1: Thymocyte differentiation antigen 1, synonym CD90
VDR: Vitamin D receptor
VPA: Valproic acid
